# A20 Is Increased in Fetal Lung in a Sheep LPS Model of Chorioamnionitis

**DOI:** 10.1155/2022/6421419

**Published:** 2022-01-20

**Authors:** Steffen Kunzmann, Matthias Hütten, Barbara Ottensmeier, Boris W. Kramer, Markus Fehrholz

**Affiliations:** ^1^Children's Hospital, University of Würzburg, Germany; ^2^Clinic of Neonatology, Bürgerhospital Frankfurt Am Main, Germany; ^3^Children's Hospital, University of Maastricht, Research School of Oncology and Developmental Biology (GROW), Netherlands; ^4^Monasterium Laboratory, Skin and Hair Research Solutions GmbH, Muenster, Germany

## Abstract

Chorioamnionitis is associated with an increased risk of preterm birth and aggravates adverse outcomes such as BPD. Development of BPD is associated with chronic inflammatory reactions and oxidative stress in the airways which may be antenatally initiated by chorioamnionitis. A20 is an immunomodulatory protein involved in the negative feedback regulation of inflammatory reactions and is a possible regulator protein in oxidative stress reactions. The influence of chorioamnionitis on A20 gene regulation in the fetal lung is unknown. We characterized the influence of LPS and proinflammatory cytokines on A20 expression in human lung endothelial (HPMEC-ST1.6R) and epithelial (A549) cells *in vitro* by real-time PCR and/or western blotting and used a sheep model of LPS-induced chorioamnionitis for *in vivo* studies. To study the functional role of A20, endogenous A20 was overexpressed in HPMEC-ST1.6R and A549 cells. LPS induced proinflammatory cytokines in HPMEC-ST1.6R and A549 cells. Both LPS and/or proinflammatory cytokines elevated A20 at transcriptional and translational levels. Intra-amniotic LPS transiently increased IL-1*β*, IL-6, IL-8, and TNF-*α* mRNA levels in fetal lamb lungs, associated with an increase in A20 mRNA and protein levels. Overexpression of A20 reduced proinflammatory cytokines in vitro. Repeated LPS exposure induced LPS tolerance for proinflammatory cytokines and A20 *in vitro* and *in vivo*. Antenatal inflammation induced a transient increase in proinflammatory cytokines in the preterm fetal lung. The expression of proinflammatory cytokines increased expression of A20. Elevated A20 may have a protective role by downregulating chorioamnionitis-triggered fetal lung inflammation. A20 may be a novel target for pharmacological interventions to prevent chorioamnionitis-induced airway inflammation and lung damage, which can result in BPD later in life.

## 1. Introduction

Bronchopulmonary dysplasia (BPD) is still the most common adverse outcome after preterm birth. Patients with BPD have reduced area for gas exchange which is the result of an impaired lung development in both the alveoli and the microvasculature. The disturbed development of alveoli and the microvasculature is highly associated with lung inflammation- and oxygen toxicity-induced airway and vascular remodeling [1, 2]. However, the underlying mechanisms of this disturbed lung development during chronic inflammation and oxidative stress remain unclear [3, 4]. In particular, the physiological mechanisms for the regulation of lung inflammation are less well defined, both *in vitro* and *in vivo*, with respect to resolution of the inflammatory response.

For preterm infants, pulmonary inflammation can already begin *in utero* due to chorioamnionitis, which is a microbial infection of the amnion and chorion [5]. Chorioamnionitis is one of the leading factors associated with preterm birth [6]. It has been reported that the rate of incidence of histologic chorioamnionitis is 45–60% in very low birth weight (VLBW) infants [5]. Chorioamnionitis elevates proinflammatory cytokines in human amniotic fluid and fetal cord blood, most likely in response to bacterial products and injury [7]. It is believed that such proinflammatory cytokines are mediators that recruit activated inflammatory cells to the fetal lung [3, 4]. Fetal sheep develop chorioamnionitis if LPS is injected into the amniotic fluid, initiating a sequence of lung injury consistent of inflammation, apoptosis, oxidative stress, and remodeling [8, 9]. This consequently results in lung maturation as well as decreased alveolar septation including microvascular injury [3, 10]. All of these changes may initiate a progression to BPD in the fetal lung [3, 11].

A20, which is also termed tumor necrosis factor- (TNF-) *α* induced protein-3 (TNFAIP3), is a zinc finger protein first described as the product of a TNF-*α* responsive gene in endothelial cells [12], but also expressed in a number of different cell types such as epithelial [13] or immune cells [14, 15]. Two adjacent NF-*κ*B–binding sites in the A20 promoter mediate the expression of A20, which is therefore regulated by NF-*κ*B [16]. A20 is a negative regulator of inflammation which is mediated by modulating the activity of NF-*κ*B. [17, 18]. In addition, A20 has vasculoprotective functions in an animal model of hypoxia-induced pulmonary hypertension [19]. The expression of A20 can reduce endotoxin-induced neutrophil sequestration and lung vascular leak [20]. Deubiquitinase function of A20 maintains and repairs endothelial barrier after lung vascular injury [21]. Overexpression of A20 can also inhibit cell death induced by proinflammatory cytokines and A20 knockout mice are more susceptible to TNF-*α*-stimulated cell death [22]. Increased survival of cells exposed to oxidative stress has been linked to the activation of NF-*κ*B [23]. Thus, A20 may be of potential therapeutic interest for lung disease treatments by resolving inflammation and limiting vascular injury and oxidative stress reactions [17, 19, 23, 24]. Until now, no studies were carried out to investigate the effect of chorioamnionitis on A20 expression in the fetal lung, while the role of A20 in BPD of preterm infants is also unknown.

We therefore hypothesized that antenatal inflammation would increase the expression of A20 in preterm lungs, thereby affecting the expression of proinflammatory cytokines involved in chorioamnionitis-induced lung inflammation.

## 2. Methods

### 2.1. Reagents

Lipopolysaccharide (LPS) from *Escherichia coli* serotype 055:B5, recombinant human TNF-*α* and IL-1*β* were purchased from Sigma-Aldrich (St. Louis, CA).

### 2.2. Cell Culture

HPMEC-ST1.6R, a human LEC line, has already been described and exhibited a broad spectrum of primary human microvascular endothelial cell characteristics *in vitro* [25, 26]. A549 cells, a human lung carcinoma cell line with characteristics of human alveolar basal epithelial cells, were purchased from ATCC (LGC Standards, Teddington, UK) [27].

HPMEC-ST1.6R were grown on plastic tissue culture dishes in RPMI medium (Sigma-Aldrich) containing 10% fetal bovine serum, penicillin (100 U/mL), streptomycin (100 *μ*g/mL), and amphotericin B (0.25 *μ*g/mL). A549 cells were cultured in DMEM (Sigma-Aldrich) with 5% fetal bovine serum (Gibco, Thermo Fisher Scientific), 100 U/mL penicillin, and 100 *μ*g/mL streptomycin (Sigma Aldrich). Experiments with TGF-*β*1 were performed in serum-free medium. On 6 cm dishes, cells were allowed to grow to 80% confluence before adding the investigated agents. Incubation was carried out at 37°C in a humidified atmosphere of 95% room air and 5% CO_2_.

HPMEC-ST1.6R or A549 cells were incubated with LPS (100 ng/mL), IL-1*β* (10 ng/mL), or TNF-*α* (10 ng/mL) for different times as indicated in the figures. For the tolerance experiments, cells were first exposed to LPS (100 ng/mL) for 4 h; then, LPS was washed off and after a 24 h recovery period the cells were exposed to LPS (100 ng/mL) for 4 h a second time.

### 2.3. Overexpression of A20

For the overexpression of A20, the lentiviral system as described by Zinke et al. was used [28]. The A20 open reading frame was amplified from pEGFP-C1-A20 [29] using primers NheIA20fwd 5′-CACCGCTAGCATGGCTGAACAAGTCCTTCCTCAGGC-3′ and Bsp119IA20rev 5′-CCTATTCGAATTAGCCATACATCTGCTTGAACTGAAAGC-3′ (pEGFP-C1-A20 was a kind gift from Yihong Ye (Addgene plasmid # 22141)) and inserted into pCW_EF1a_rtTA_Puro (a kind gift from Dr. David Schrama and Dr. Roland Houben, Department of Dermatology, University Hospital Wuerzburg). The correct sequence of the construct was verified by sequencing. Vesicular stomatitis virus envelope protein G (VSV-G)-pseudotyped lentiviral particles were produced by transfection of 293T cells with plasmids pMDLg, pRSV-Rev, and pMD.G as described previously [28]. Sterile-filtered particles were further concentrated using 100 kDa Amicon Ultra-15 filters (Merck Millipore, Billerica, MA). After transduction with A20-expressing lentiviral vectors, A549 and HPMEC-ST1.6R cells were expanded in culture medium containing 2 *μ*g/mL puromycin. Expression of A20 mRNA in transduced cells was induced using 1 *μ*g/mL doxycycline. Noninduced cells were used as control.

### 2.4. Animals, Intra-Amniotic Injections, and Tissue Processing at Delivery

The chorioamnionitis sheep model used in this study has been described previously [30, 31]. In brief, all animals were studied in Western Australia with approval from the Institutional Animal Care and Use Committees of the Cincinnati Children's Hospital (Cincinnati, OH), and the Western Australian Department of Agriculture (Animal Ethics Committee (reference number RA/3/100/312)). Time-mated Merino ewes with singleton fetuses were randomly assigned to groups of five to nine animals, to receive either a single injection of 10 mg of LPS (*Escherichia coli* 055:B5; Sigma-Aldrich) (*n* = 7), two injections of 10 mg of LPS (*n* = 7), or an equivalent volume of saline (control) by intra-amniotic injections for intervals of 2 or 7 days (or 2 and 7 days) (*n* = 7) before caesarean delivery at 124 ± 1 days gestational age. The control fetal lambs given one or two injections of intra-amniotic saline were combined because there were no differences in the measurements between the single vs. double injections of saline (*n* = 6). Intra-amniotic injections were given under ultrasound guidance with verification of needle placement by electrolyte analysis of the amniotic fluid aspirated immediately before injection. Pieces of the right lower lobe of the lung were snap-frozen for RNA analysis.

### 2.5. RNA Extraction and Reverse Transcription

Total RNA was isolated from tissue from the right lower lung lobe by guanidinium thiocyanate-phenolchloroform extraction, as described previously [30]. Total RNA of HPMEC-ST1.6R or A549 cells was isolated using NucleoSpin® RNA Kit (Macherey-Nagel, Dueren, Germany) according to the manufacturer's protocol. Total RNA was eluted in 60 *μ*L of nuclease-free H_2_O (Sigma-Aldrich) and stored at -80°C until reverse transcription. For reverse transcription PCR, 1 *μ*g of total RNA was reverse transcribed using the High-Capacity cDNA Reverse Transcription Kit (Applied Biosystems, Thermo Fisher Scientific) according to the manufacturer's instructions. Upon analysis, first-strand cDNA was stored at -20°C.

### 2.6. Real-Time PCR Analysis

For detection of human (h) and sheep (ovine (ov)) IL-1*β*, IL-6, IL-8, TNF-*α*, A20, and *β*-actin mRNA, cDNA was analyzed using 12.5 *μ*L iQ™ SYBR® Green Supermix (Bio-Rad Laboratories, Hercules, CA), 0.5 *μ*L deionized H_2_O, and 10 pmol each of forward and reverse primers. Primers for the detection of IL-1*β*, IL-6, IL-8, TNF-*α*, A20, and *β*-actin mRNA are shown in Table 1.

Real-time PCR was performed on an ABI Prism 7500 Sequence Detection System (TaqMan®) as described [32]. Melt curve analyses were performed to verify single PCR products. Results were normalized to *β*-actin, and mean fold changes in mRNA levels were calculated by the *ΔΔ*C_T_ method by Livak and Schmittgen [33]. Experiments were carried out in duplicate and repeated at least three times.

### 2.7. Western Blot Analysis

Western blot analysis from frozen lung tissue was performed as previously described [30]. HPMEC-ST1.6R or A549 cells were rinsed with ice-cold tris-buffered saline (TBS) and incubated in 100 mL lysis buffer (Cell lysis buffer, Cell Signaling Technologies, MA, USA, cOmplete Mini protease inhibitor cocktail tablets and PhosStop phosphatase inhibitor cocktail tablets (Roche, Germany; 0.1 mM PMSF, Merck KGaA, Germany)) for 10 min on ice. The lysate was cleared by centrifugation at 30,000 × g for 10 min, and the supernatant was used for western immunoblotting analysis. Protein concentrations were determined for each sample using the Bradford assay (Bio-Rad, Richmond, CA, USA), and equal amounts of cellular protein were loaded and separated by SDS-PAGE on 10% to 12% Bis-Tris gels and electrophoretically transferred to polyvinylidene difluoride blotting membranes (Amersham Pharmacia Biotech, Piscataway, NJ, USA). Membranes were blocked in 5% BSA for 1 h at room temperature and successively incubated with primary antibodies overnight at 4°C. Blots were probed with primary antibodies to *β*-actin (926-42212; LI-COR Inc., Lincoln, NE, USA; dilution 1 : 1000) or A20 (ab93868; Abcam, Cambridge, United Kingdom; dilution 1 : 5000), followed by the corresponding horseradish peroxidase-conjugated secondary antibody (Pierce, Bonn, Germany) for 1 h at room temperature. Specific protein bands were visualized using Clarity™ Western ECL Substrate (Bio-Rad Laboratories, Hercules, CA) and a ChemiDoc™ MP Imaging System (Bio-Rad Laboratories). Captured signals were quantified by densitometric analysis using Image Lab™ Software v5.2.1 (Bio-Rad Laboratories).

### 2.8. Data Analysis

Results are given as means ± SD. Data were analyzed using one-way ANOVA with Sidak's multiple comparisons test or Student's *t*-test. A *p* value ≤ 0.05 was considered significant. All statistical analyses were performed using Prism® version 6 (GraphPad Software, San Diego, CA).

## 3. Results

### 3.1. Effect of LPS on Proinflammatory Cytokine Production in Different Lung Cell Lines

We first examined the effects of LPS on proinflammatory cytokine production in different lung cell culture lines. After 4 h incubation, LPS increased mRNA expression of IL-1*β* (4.6-fold), IL-6 (100-fold, *p* < 0.05), IL-8 (85-fold, *p* < 0.05), and TNF-*α* (26-fold) in human lung endothelial cells (HPMEC-ST1.6R) (Figure 1(a)). In lung epithelial cells (A549) the response of LPS on proinflammatory cytokine production was lower (IL-1*β* (3.0-fold), IL-6 (2.2-fold), IL-8 (7.8-fold, *p* < 0.05), and TNF-*α* (5.6-fold)) compared to HPMEC-ST1.6R (Figure 1(b)).

These results indicate that LPS increases proinflammatory cytokine production at the transcriptional level to a different extent in different lung cell lines.

### 3.2. Effect of LPS and Proinflammatory Cytokines on A20 Production in Different Lung Cell Lines

We examined the effects of LPS and proinflammatory cytokines on A20 expression in human lung endothelial cells (HPMEC-ST1.6R) and lung epithelial cells (A549). In human lung endothelial cells (HPMEC-ST1.6R), we found a significant transient increase in A20 mRNA levels by LPS with a maximal 20-fold increase after 4 h (16 h: 1.9-fold, 24 h: 1.8-fold). For TNF-*α*, only a moderate effect on A20 expression could be detected in HPMEC-ST1.6R cells (4 h: 4.3-fold, 16 h: 4.5-fold, 24 h: 5.3-fold), while IL-1*β* showed negligible effects on A20 expression (4 h: 1.5-fold, 16 h: 0.8-fold, 24 h: 1.5-fold) (Figure 2(a)). At the translational level, we found a nonstatistic significant “increase” of A20 synthesis by LPS, IL-1*β*, and TNF-*α* after 12 and 24 h (Figure 2(b)).

In lung epithelial cells (A549), we found an increase of A20 mRNA levels by IL-1*β* (4 h: 42-fold, 16 h: 14-fold, 24 h: 13-fold) and TNF-*α* (4 h: 51-fold, 16 h: 58-fold, 24 h: 20-fold), while no effect of LPS could be detected (Figure 2(c)). At the translational level, we confirmed the effect of IL-1*β* and TNF-*α* on A20 protein synthesis after 12 h, 24 h, and 48 h (Figure 2(d)).

Taken together, these data show that LPS induces an early and transient induction of A20 mRNA in HPMEC-ST1.6R cells and that the proinflammatory cytokines IL-1*β* and TNF-*α* can induce A20 mRNA and protein expressions for a longer time in A549 cells, while LPS has no effect on A20 expression.

### 3.3. Effects of Repeated LPS Exposure on Proinflammatory Cytokine and A20 mRNA Levels in Lung Endothelial Cells

To determine whether preincubation of HPMEC-ST1.6R cells with LPS may influence the observed effect of LPS on proinflammatory cytokine and A20 expression, HPMEC-ST1.6R cells were preincubated with LPS before the cells were stimulated a second time with LPS for 4 h. In double-stimulated cells, no induction of IL-1*β*, IL-6, IL-8, TNF-*α*, or A20 mRNA expressions could be observed (Figure 3 right (white columns)) while single stimulated cells showed significant induction of IL-6 (47-fold, *p* < 0.05), IL-8 (40-fold, *p* < 0.05), TNF-*α* (46-fold, *p* < 0.05), and A20 (20-fold, *p* < 0.05) (Figure 3 left (black columns)).

In conclusion, repeated LPS exposure can inhibit single LPS-induced proinflammatory cytokine and A20 mRNA levels in lung endothelial cells.

### 3.4. Effects of Single and Repeated Intra-Amniotic LPS on Proinflammatory Cytokine mRNA Expression in Fetal Sheep Lung

To confirm our *in vitro* results *in vivo*, we measured proinflammatory cytokine production in fetal lungs in a chorioamnionitis sheep model. The mRNAs of proinflammatory cytokines were induced in the fetal lung, displaying maximum levels after 2 days following single intra-amniotic LPS exposure (IL-1*β* (197-fold), IL-6 (23-fold), IL-8 (29-fold), and TNF-*α* (5-fold)). Lower induction was observable 7 days after exposure to a single injection of intra-amniotic LPS (IL-1*β* (31-fold), IL-6 (3.5-fold), IL-8 (25-fold), and TNF-*α* (2.4-fold)) (Figure 4). In contrast, a prior exposure to intra-amniotic LPS 7 days before delivery inhibited the induction of IL-1*β*, IL-6, IL-8, and TNF-*α* mRNA levels after intra-amniotic LPS challenge was administered 2 days before delivery (intra-amniotic LPS 2- plus 7-day group).

In summary, intra-amniotic LPS (single injection) induced proinflammatory cytokine expression in the fetal lung at 2 days, with lower values 7 days after exposure. Repeated intra-amniotic LPS injections did not induce proinflammatory cytokine mRNA suggesting LPS-tolerance.

### 3.5. Effects of Intra-Amniotic LPS on A20 Expression in Fetal Sheep Lung

To study the effects of intra-amniotic LPS on the expression of A20 in the fetal lung, we analyzed A20 mRNA and protein levels. A20 mRNA level was increased 12-fold in the fetal lung at 2 days with a reduction by 7 days (3.5-fold) after exposure to a single injection of intra-amniotic LPS (Figure 5(a)). To confirm that the increased level of A20 mRNA corresponded with enhanced protein concentrations, A20 was quantified by western blot analysis. A20 protein synthesis was increased at 2 days with a reduction to control levels by 7 days after a single injection of intra-amniotic LPS (Figure 5(b)). A20 mRNA and protein expression in lungs of fetal lambs exposed to repeated intra-amniotic LPS (2 plus 7-day group) was like those seen in the control group (Figures 5(a) and 5(b)).

Taken together, LPS-induced chorioamnionitis induces a transient A20 expression on mRNA and protein level, while repeated intra-amniotic LPS inhibits A20 expression in the fetal lung.

### 3.6. Effects of A20 Overexpression on LPS-Induced Proinflammatory Cytokine Production in Human Lung Endothelial (HPMEC-ST1.6R) and A549 Cells

The expression of A20 has been reported to involve the negative feedback regulation of TNF-*α*-induced NF-*κ*B-dependent gene expression [16]. We therefore hypothesized that the LPS-mediated induction of A20 may function as a negative feedback loop of TLR-4 signaling. To address this issue, we studied the effects of overexpressing A20 in HPMEC-ST1.6R and A549 cells on LPS-mediated proinflammatory cytokine induction, using real-time PCR.

Overexpression of A20 was confirmed by real-time PCR and western blot analysis in HPMEC-ST1.6R (Figure 6(a)) and A549 cells (Figure 6(c)). Overexpression of A20 in HPMEC (Figure 6(b)) and A549 (Figure 6(d)) significantly inhibited NF-*κ*B-dependent IL-6, IL-8, and TNF-*α* gene expressions induced by LPS.

Taken together, overexpression of A20 significantly diminished LPS-induced proinflammatory cytokine production in human lung endothelial (HPMEC-ST1.6R) and A549 epithelial cells.

## 4. Discussion

In this study, we describe for the first time an antenatal transient upregulation of A20 in the fetal sheep lung induced by chorioamnionitis. *In vitro*, we confirmed the upregulation of A20 by LPS itself and/or the two proinflammatory cytokines IL-1*β* and TNF-*α* in lung endothelial and epithelial cell lines, respectively. Beside IL-6, IL-8, IL-1*β*, and TNF-*α* mRNA levels were also upregulated in the fetal lung after intra-amniotic LPS exposure. Repeated LPS exposure induced LPS tolerance *in vivo* and *in vitro* by inhibiting proinflammatory cytokine and A20 induction. Overexpression of A20 in these two cell lines inhibited the LPS-triggered proinflammatory cytokine response, underlining the anti-inflammatory effects of A20 in different lung cell types. The results may suggest that during chorioamnionitis, A20 functions as a negative regulator of airway inflammation by counteracting proinflammatory cytokine synthesis induced by LPS. Chorioamnionitis-induced A20 expression could be thus an endogenous feedback mechanism to switch off or limit an initial inflammatory reaction in the lung which might have positive effects by minimizing inflammation-induced lung damage in chorioamnionitis.

The blood-air barrier is formed by lung microvascular endothelial and alveolar epithelial cells, and its disruption is a hallmark of acute lung injury [34]. Lung epithelial cells form an important site for innate immune responses, functioning as a primary interface between pathogens and the airway. The airway epithelium is a major player in the mucosal immune response, which is able to express proinflammatory cytokines and to recruit inflammatory cells in response to pathogenic bacteria [35, 36]. Besides the airway epithelium, vascular endothelial cells play an important role in many pathologies, including inflammation, oxidative stress, vascular remodeling, and thrombosis [37]. In combination with a disturbed integrity of the lung's alveolar-capillary, these processes are involved in chorioamnionitis-induced lung damage [3, 38]. For this reason, lung epithelial and endothelial cell lines were chosen for our study.

As a first step, we characterized the effects of LPS on the induction of proinflammatory cytokines in these two lung cell lines. While an early and strong effect of LPS on the mRNA synthesis for the proinflammatory cytokines IL-1*β*, IL-6, IL-8, and TNF-*α* was observed in HPMEC-ST1.6R cells, only minor effects of LPS in A549 cells were visible. We assumed that both cell lines—lung endothelial (HPMEC-ST1.6R) and epithelial cells (A549)—would respond profoundly to LPS, especially since the response in primary epithelial cells has already been reported [39]. However, considerable differences in cytokine response between A549 cells and primary alveolar epithelial cells type II (AEC-II) are described [39]. The epithelial cells may be more frequently exposed to pathogens which may explain the reduced response (immunoreactivity) in comparison to the endothelial cells.

In parallel, in our *in vivo* system, intraamniotic LPS increased the proinflammatory cytokines IL-1*β*, IL-6, IL-8, and TNF-*α* in the fetal sheep lung. This is consistent with other previous studies, in which the mRNAs for proinflammatory cytokines were induced in the fetal lung after intra-amniotic LPS exposure [31, 40].

It has been suggested that the mechanisms that downregulate inflammatory responses in the innate immunity of airway epithelium and endothelium may play important roles in controlling inflammatory lung diseases [41]. During inflammation and infection, these regulators may contribute to limiting proinflammatory cytokines. One of these regulators is A20, encoded by an immediate early-response gene and acting as an inhibitor of NF-*κ*B-dependent gene expression. A20 is induced independently by different stimuli including LPS [42], TNF-*α*, or IL-1*β* [43]. LPS-induced expression of A20 has already been reported in primary human airway epithelial cells [41]. Our current results confirmed these findings in a chorioamnionitis animal model and in an *in vitro* lung cell system. LPS induced only a transient A20 mRNA induction in the lung endothelial cell line HPMEC-ST1.6R, while no effect of LPS could be observed in the lung epithelial cell line A549. However, in contrast to LPS, IL-1*β* and TNF-*α* induced an A20 expression on mRNA and protein level in A549 cells, which was stronger and for a longer duration compared to HPMEC-ST1.6R cells. This robust A20 induction in lung epithelial cells could be responsible for a reduced immunoreactivity of epithelial cells as primary contact cells with pathogens in the lung.

We demonstrated for the first time that intra-amniotic LPS-induced increased levels of A20 mRNA and protein in the fetal sheep lung. The LPS is administered to the amniotic fluid and reaches the fetal via the fetal airways. Until now, the regulation of A20 in TLR-mediated inflammation in chorioamnionitis has not been characterized in detail. *In vivo*, a “cocktail” of certain stimuli including bacterial LPS, as a primary and early stimulus, as well as pro-inflammatory, airway-cell-produced cytokines like IL-1*β* and TNF-*α* as a secondary stimulus, could be responsible for the synthesis of A20 in the lung in the chorioamnionitis model.

Furthermore, our results confirm LPS tolerance (alternative names: endotoxin hyporesponsiveness/immunoparalysis) for LPS-induced proinflammatory cytokine expression in our *in vitro* and *in vivo* test system. This observation confirms that LPS-tolerance induced by exposure to inflammation *in utero* may prevent fetal lung damage by a prolonged inflammatory reaction [31, 44]. Besides proinflammatory cytokines, we report for the first time LPS tolerance for induction of A20 after repeated LPS exposures *in vitro* and *in vitro*.

Dysregulation of A20 has been described in various lung diseases and lung models. For instance, A20 is reduced basally and after LPS stimulation in cystic fibrosis airway epithelial cells [45]. In addition, a reduction of A20 has been associated with markers of inflammation and decreased lung function [13]. In contrast, in mouse models for asthma, it was shown that A20 overexpression had protective effects with regard to airway inflammation and normalized the inflammatory response in airways [24]. In a rat model of acute lung injury, LPS upregulated A20, modulating the immune response by downregulation of NF-*κ*B and macrophage polarization [46]. Furthermore, in a hypoxia-induced pulmonary artery hypertension animal model, A20 deficiency led to angiogenesis of pulmonary artery endothelial cells through elevated NF-*κ*B activation in hypoxia [19]. Our study adds that A20 is transiently upregulated in the fetal lung in a chorioamnionitis sheep model and part of the regulated proteins in endotoxin tolerance.

To further characterize the functional role of an overexpression of A20 in the lungs of LPS-exposed lambs, we explored the pulmonary anti-inflammatory effects of A20 in lung endothelial and epithelial cells *in vitro*. We demonstrated that overexpression of A20 had the ability to inhibit LPS-induced NF-*κ*B-dependent gene expression of proinflammatory cytokines IL-1*β*, IL-6, IL-8, and TNF-*α* in both HPMEC-ST1.6R and A549 cells. O'Reilly and colleagues have previously reported that A20 abolished TLR-4 activation of NF-*κ*B in HEK293 cells cotransfected with TLR4 [47]. Our results confirm the role of A20 in modulating LPS induced inflammation which is in line with the phenotype of A20^−/−^ mice that are highly susceptible to LPS. In addition, in primary epithelial airway cells, the overexpression of A20 inhibited the activation of both NF-*κ*B and IL-8 promoter activity [41]. Thus, in our chorioamnionitis model, A20 may regulate TLR-induced airway inflammation accompanied by a reduction of IL-1*β*, IL-6, IL-8, and TNF-*α*. These cytokines are well known to contribute to excessive airway inflammation. Therefore, modulating an overproduction of these proinflammatory cytokines may attenuate airway inflammation [48].

In addition to its modulatory part in airway inflammation, a functional role of A20 in airway vascular injury has been postulated [19, 49], which is in line with our findings in an endothelial cell line. A20 attenuated hypoxia-induced pulmonary arterial hypertension by inhibiting NF-*κ*B activation and pulmonary artery smooth muscle cell proliferation [19, 49]. A transient elevation of A20 was found in lung tissues from hypoxic rats compared with normoxic controls [19, 49]. This rapid enhancement was mainly detected in the endothelium. During early hypoxia, genetic inhibition of A20 increased proliferation in pulmonary artery endothelial cells [19, 49]. Furthermore, A20 maintains and repairs endothelial barrier after lung vascular injury [21]. The deubiquitinase function of endothelial A20 is required to maintain and repair the endothelial barrier after inflammatory lung vascular injury through VE-cad (vascular endothelial cadherin) expression at endothelial adherent junctions [21].

In addition, overexpression of A20 can inhibit cells death induced by inflammatory cytokines [50]. A20 can thus prevent TNF-*α*-induced cell cytotoxicity by inhibiting both TNF-*α*-induced apoptosis and necrosis [50]. Despite its antiapoptotic function in cytokine signaling, A20 can enhance death mediated by oxidative stress [51].

The exact role of A20 in vascular remodeling and in cytokine-/oxidative-stress mediated cell death in our chorioamnionitis model is studied in the moment.

These results indicate that A20 functions as a negative regulator of airway inflammation by counteracting the activation of TLR-4 by LPS. Thus, A20 might play a critical role in limiting chorioamnionitis-triggered inflammation by terminating TLR-induced NF-*κ*B responses in the airway and endothelial cells. Hence, the endogenous molecule A20 could be a key target to control or normalize the inflammatory response-induced antenatally in the lung by chorioamnionitis. A20 regulation could be a new target for pharmacological interventions against BPD development which is the result of inflammatory changes on both sides of the blood-air barrier.

## Figures and Tables

**Figure 1:** LPS-induced proinflammatory cytokine production in different lung cell lines. HPMEC-ST1.6R (Figure 1(a)) and A549 cells (Figure 1(b)) were incubated with LPS (100 ng/mL) for 4 h. mRNA levels of IL-1*β*, IL-6, IL-8, and TNF-*α* normalized to *β*-actin mRNA levels were measured by real-time PCR. Means + SD of *n* = 3 independent experiments are shown. ^∗^*p* < 0.05 compared to untreated cells.

**Figure 2:** LPS- and proinflammatory cytokine-induced A20 expression in different lung cell lines. HPMEC-ST1.6R (a, b) and A549 cells (c, d) were incubated with or without LPS (100 ng/mL), IL-1*β* (10 ng/mL), or TNF-*α* (10 ng/mL) for the indicated time. Real-time PCR of A20 mRNA was performed after 4 h, 16 h, or 24 h (a, c) and western blot analysis was carried out after 12 h, 24 h, or 48 h (b, d). Relative mRNA (protein) levels of A20 were calculated by normalizing signals to detected *β*-actin mRNA (protein). Differences compared to untreated cells were calculated. Means + SD of *n* = 3 independent experiments are shown. (b, d) Representative immunoblots of *n* = 3 independent experiments are shown. ^∗^*p* < 0.05 compared to control cells.

**Figure 3:** Repeated LPS exposure inhibits single LPS-induced proinflammatory cytokine and A20 mRNA expressions in HPMEC-ST1.6R cells. HPMEC-ST1.6R cells were incubated with LPS (100 ng/mL) for 4 h (A, black column) or cells were first exposed to LPS (100 ng/mL) for 4 h, then LPS was washed off and after a 24 h recovery period the cells were exposed to LPS (100 ng/mL) for 4 h a second time (B, white column). mRNA levels of IL-1*β*, IL-6, IL-8, TNF-*α*, and A20 were measured by real-time PCR and normalized to *β*-actin mRNA level. Means + SD of *n* = 3 independent experiments are shown. ^∗^*p* < 0.05 compared to untreated cells, ^#^*p* < 0.05 compared to respective 4 h single treated cells.

**Figure 4:** Effects of intra-amniotic LPS on proinflammatory cytokine mRNA levels in the fetal sheep lung. Chorioamnionitis was induced by an ultrasound-guided injection of LPS from *E. coli* into the amniotic fluid of singleton, time-mated pregnant sheep. Quantification of IL-1*β* (a), IL-6 (b) IL-8 (c), or TNF-*α* mRNA (d) from the fetal sheep lung normalized to *β*-actin. The mean mRNA signal in control animals was given the value of 1, and levels at each time point were expressed relative to controls. Means + SD of *n* = 3 independent experiments are shown. ^∗^*p* < 0.05 versus control, ^#^*p* < 0.05 versus single LPS 2-day exposure.

**Figure 5:** Intra-amniotic LPS-induced A20 mRNA and protein expression in the fetal sheep lung. Chorioamnionitis was induced by an ultrasound-guided injection of LPS from *E. coli* into the amniotic fluid of singleton, time-mated pregnant sheep. (a) Quantification of A20 mRNA from the fetal sheep lung was normalized to *β*-actin. The mean mRNA signal in control animals was given the value of 1, and levels at each time point were expressed relative to controls. (b) A representative immunoblot of *n* = 3 independent experiments is shown. Concentrations of A20 and *β*-actin protein were semiquantified by densitometry. Optical density of A20 protein band was corrected to *β*-actin, and mean value in control animals was given the value of 1, and levels at each time point were expressed relative to controls. Means + SD of *n* = 3 independent experiments are shown. ^∗^*p* < 0.05 versus control, ^#^*p* < 0.05 versus single LPS 2-day exposure.

**Figure 6:** A20 overexpression inhibits LPS-induced proinflammation cytokine expression in HPMEC and A549 cells. (a, c) Detection of A20 overexpression in HPMEC-ST1.6R (a) and A549 (c) cells. A20 mRNA and protein were detected by real-time PCR (lower part) and western blot analysis (upper part). (b, d) HPMEC-ST1.6R (b) and A549 (d) cells transduced with A20-expressing retroviral vectors. A20 expression was induced by doxycycline (white bars) and cells were stimulated with LPS (100 ng/mL) for 4 h. Real-time PCR for IL-1*β*, IL-6, IL-8, and TNF-*α* was performed. Means + SD of *n* = 3 independent experiments are shown. ^#^*p* < 0.05, compared to respective LPS-stimulated cells without doxycycline (black bars).

**Table 1:** RT-PCR primers.

Primer name	Primer sequence	Accession number
hIL-1*β*fwd	5′-TTCATTGCTCAAGTGTCTG-3′	NM_000576.3
hIL-1*β*rev	5′-GCACTTCATCTGTTTAGGG-3′	NM_000576.3
ovIL-1*β*fwd	5′-CCTGTCATCTTCGAAACATCC-3′	NM_001009465.2
ovIL-1*β*rev	5′-GCAGAACACCACTTCTCGG-3′	NM_001009465.2
hIL-6fwd	5′-CTCTCATTAAGCACATCGT-3′	NM_001009392.1
ovIL-6rev	5′-GATCAAGCAAATCGCCTG-3′	NM_001009392.1
hIL-8fwd	5′-CAGTGCATAAAGACATACTCC-3′	NM_000584.4
hIL-8rev	5′-TTTATGAATTCTCAGCCCTC-3′	NM_000584.4
ovIL-8fwd	5′-AAACACATTCCACACCTTTCC-3′	NM_001009401.2
ovIL-8rev	5′-GGATCTTGCTTCTCAGCTCTC-3′	NM_001009401.2
hTNF-*α*fwd	5′-CAGCCTCTTCTCCTTCCT-3′	NM_000594.4
hTNF-*α*rev	5′-GGGTTTGCTACAACATGG-3′	NM_000594.4
ovTNF-*α*fwd	5′-ACACTCAGGTCATCTTCTC-3′	NM_001024860.1
ovTNF-*α*rev	5′-GGTTGTCTTTCAGCTCCA-3′	NM_001024860.1
hA20fwd	5′-GCACGCTCAAGGAAACAG-3′	NM_001270507.2
hA20rev	5′-CCAGTTCCGAGTATCATAGCA-3′	NM_001270507.2
ovA20fwd	5′-AACAAATGGTGACGGAAACTG-3′	XM_027972494.2
ovA20rev	5′-GTGTCGTAGCAAAGCCCA-3′	XM_027972494.2
h*β*-actinfwd	5′-AAGATCAAGATCATTGCTCC-3′	NM_001101.5
h*β*-actinrev	5′-CTAAGTCATAGTCCGCCT-3′	NM_001101.5
ov*β*-actinfwd	5′-ATCTGTCGTCAGCAGGTC-3′	NM_001009784.3
ov*β*-actinrev	5′-CCAACGGTACTGAGAGGA-3′	NM_001009784.3

## Data Availability

Data is available within the article.
